# Preparation and Performance Analysis of Transformer Aramid Nanopaper-Based Insulating Material Based on Deep Learning

**DOI:** 10.1155/2022/2282870

**Published:** 2022-08-11

**Authors:** Bowen Liu, Fangcheng Lv, Xiaozhou Fan, Yueyi Sui, Jiaxue Wang, Shengdong Yin

**Affiliations:** ^1^Hebei Provincial Key Laboratory of Power Transmission Equipment Security Defence, North China Electric Power University, Baoding 071003, Hebei, China; ^2^State Key Laboratory of Alternate Electrical Power System with Renewable Energy Sources, North China Electric Power University, Beijing 102206, China; ^3^Ganzhou Longbang Material Technology Co., Ltd, Ganzhou 341000, Jiangxi, China

## Abstract

Transformers are an essential part of power production. Insulating paper began to be widely used in transformers in the 1990s. The superior aramid nanofiber as the matrix gives the aramid nano-insulating paper excellent mechanical properties, insulation performance, temperature resistance, and flexibility. At first, the heat resistance and service life of insulating paper should be satisfied for use in electrical equipment. With the continuous development of power equipment, people have put forward higher requirements on the properties of insulating paper, especially heat resistance and electrical properties. Insulation paper made of aramid fibers have better thermal stability and more advantages in electrical and mechanical properties, which can significantly improve the service life and safety of electrical appliances. The purpose of this article is to study the use of aramid nanopaper-based insulating materials in transformers to explore the effect of transformer discharge mechanism on aramid nanopaper-based insulating materials. This paper proposes to design multiple deep learning models to identify the discharge mode of the voltage transformer, find the characteristic signal, and carry out related tests on the discharge signal of different modes, and find the maximum temperature value of the aramid nanopaper-based insulating material for industrial use. The experimental results in this paper show that the aramid nanopaper-based insulating material can be used in transformers discharge detection well, and the safety rate is increased by 20%.

## 1. Introduction

Transformers are widely used in today's production and life, whether in power plants, substations, or in transmission lines, distribution networks and many users' household equipment, they are inseparable from it. Thermal conductivity is one of the most important thermal and hygroscopic physical parameters of building materials, which is closely related to building energy consumption, indoor environment, and many other thermal and hygroscopic processes. As one of the key equipment for power operation, oil-immersed power transformers are related to the safe, stable, and effective operation of electricity. When the transformer power supply fails, it will have a destructive impact on the line, the regional power grid, and the high-efficiency power grid, so it is very important to ensure its smooth operation. Nowadays, the scale of the transformer industry has grown rapidly, and its technology and related industries have also accelerated development. The capacity of the potential rheostat has expanded from 1.4 kVA to 1000 MVA or more to meet user needs. Today, the transformation and upgrading of power systems in countries around the world are changing every day, and the capacity and voltage levels of transformers need to be transformed and upgraded. The key to upgrading the transformer capacity and voltage level is the insulation performance of the transformer. The internal insulation of the oil-immersed power transformer is composed of mineral insulation and insulating porous paper. The mineral insulating oil plays the role of insulation, cooling, arc extinguishing, and fault characteristic display during the operation of the transformer; the insulating porous paper is used as mechanical support windings, maintaining the power flow between flexibility, high strength, and unlimited strength. As shown in Figure 1, during operation, due to the influence of factors such as electric field, heat, moisture, and mechanical force, the insulation of oil paper will gradually decrease, and finally the transformer will fail due to insulation failure. In recent years, the number of transformer failures caused by corrosive sulfides has been increasing. Most of these accidents have occurred in transformers and reactors with large capacity, high strength, heavy load, and high oil temperature. The test results show that most of them are caused by insulation problems. Therefore, to improve the insulation capacity of power transformer and to ensure the insulation effect has become the primary goal of power transformer design.

Experts and scholars at home and abroad have carried out a series of studies on how to improve the insulation capacity of power transformers. Kumari et al. [1] introduced a case study of a solar power plant in Gujarat to find out the impact of photovoltaic (PV) penetration rate on transformer performance over a 1-year time span. It was found that the main reason for the change in transformer performance when solar panels are present is related to inverter, used to supply power to linear loads. Due to the voltage and current harmonics, the windings and iron cores of the transformer will have a higher temperature rise, resulting in additional losses [1]. Hussain et al. [2] studied the dielectric properties of new ester oil-based magnetic nanofluids with different nanoparticles under different electrical stress conditions, in order to optimize the properties of the prepared nanofluids by changing the concentration of nanoparticles [2]. Przybylek [3] proposed a new method for measuring the moisture of solid materials using near-infrared spectroscopy. Measure the absorbance of near-infrared waves passing through methanol and then extract water from substances in methanol. The quality of the water extracted from the sample was determined depending on the absorbance according to the concentration of water in methanol. The determined water mass to dry mass ratio of the sample allows calculation of the water percentage of the material under study. This new method of water content measurement is to determine the water content in the fiber electrical insulation material of power transformers [3]. Goulouti et al. [4] had developed a new thermal circuit breaker composed of highly insulating aramid and glass fiber reinforced polymer (AFRP and GFRP) components and aerogel particle insulation materials, and conducted experimental research on the first prototype of a load-bearing component. The use of AFRP can achieve excellent thermal performance, with linear thermal transmittance values below 0.15 W/mK [4]. Zha et al. [5] adopted a self-designed oxygen-kerosene ablation system, and proposed an ablation test method for testing the thermal structure and material ablation performance of the solid duct rocket (SDR) secondary combustion chamber. This method requires the first non-particle erosion of the silicone rubber insulating material, and then, the particle erosion experiment with the aid of alumina to analyze the erosion of the microscopic morphology of the surface of the material by the particles. The experimental structure suggests that compared with the material without particle erosion, the average burning speed of the particle eroded material is significantly faster, and the ceramic layer around the sample is destroyed, while the matrix, particle filler, and aramid fiber around the rubber carbon fiber will be destroyed. The flame oxidation peeling proves the strong erosion and destruction effect of the particles on the insulation [5]. Tra et al. [6] found that dissolved gas analysis (DGA) of insulating oil in power transformer can provide valuable information related to failures. Through his research, he concluded that the adaptive oversampling method of unbalanced data improves the diagnostic performance of power transformer [6]. D'Alessandro et al. [7] found that the influence of water content on the thermoacoustic performance of insulating materials is a subject that deserves special attention. His investigation concluded that the different responses of insulating materials to water absorption mainly depend on their source and structure. If placed in a high-humidity environment, the insulating material may absorb part of the water vapor in the air [7]. Zhang et al. [8] studied the direct current conductivity and breakdown strength of thermoplastic linear low-density polyethylene (LLDPE)/high-density polyethylene (HDPE) blends in the temperature range of 30 to 90°C. The results showed that the blends that exhibited DC performance has better temperature stability. Compared with XLPE, it shows lower conductivity and higher breakdown strength [8]. The appeal research has certain merits for improving the performance of transformers, but there are always shortcomings in actual implementation and application.

In this paper, by studying the relevant properties of aramid nanopaper-based insulating materials, and creatively combining aramid nanopaper-based insulating materials with transformers, the insulation ability of transformers is guaranteed. Based on the principle of transformer aging and discharge, a deep learning mode is introduced, and the discharge point of the transformer can be better found by constructing a voltage transformer discharge recognition model to solve the partial discharge problem of the transformers.

## 2. Transformer Discharge Identification Method and Insulation Protection Principle

### 2.1. Transformer Insulation Analysis

Insulation faults of power transformer can be divided into two categories: internal causes and external causes. The internal causes can be divided into main insulation and longitudinal insulation. External causes can be divided into electrical excursions and insulation aging. Therefore, the following three aspects of performance should be considered to solve the insulation problem of power transformers [9, 10]:

#### 2.1.1. Electrical Performance

Power transformer will be affected by two different voltages during operation, and they will damage the voltage transformer. One is the common operating voltage in daily life. This voltage is less destructive and is not common in power transformer failures. The other is a random overload voltage. This voltage has a high probability of destroying the power transformer and has a high probability of occurrence. Therefore, solving the overload voltage of the transformer is the key to ensuring the insulation capability of the transformer.

#### 2.1.2. Mechanical Properties

According to the principle of electromagnetics, in the normal working state, the transformer will flow current, and the current will generate electromotive force under the electromagnetic effect. This electric power will affect the internal performance of the power transformer. Especially when a transient short-circuit fault occurs, a large amount of current flows through the circuit at this time, generating a strong electromotive force, which will destroy the transformer very quickly and cause a fault. Therefore, we must pay attention to the impact of electric power on the transformer when designing, and select suitable insulating materials to improve the mechanical strength of the transformer.

#### 2.1.3. Thermal Performance

During the operation of the power transformer, due to the friction of the equipment, energy loss and heat loss will inevitably occur. This part of the loss will always exist during the operation of the transformer, and the continuous high temperature will damage the insulating material of the transformer, and the insulating material will gradually age and fail. Different insulating materials have different insulation levels. Although the industry has established the working temperature and maximum temperature of power transformer according to the insulation level, it is still necessary to avoid the heating temperature exceeding the maximum working temperature during actual use, otherwise the service life of the transformer will be reduced.

Industrial progress is accelerating, and transformer operation requirements are getting higher and higher, so the corresponding insulation standards are also increasing. Insulating materials need to meet the following requirements: first, the voltage value should be high enough and have good electrical properties; second, the mechanical strength should be large, and the internal should be able to withstand greater mechanical force, and the third is that the material should have strong heat resistance to minimize the heat loss of the voltage device.

### 2.2. Introduction to Dielectric Parameters

#### 2.2.1. Polarization of Dielectric

Dielectric polarization is a phenomenon in which a dielectric exhibits electrical properties under the action of an applied electric field. First of all, provide a vacuum and airtight space. In this space, apply a DC voltage of U to both ends of the plate capacitor. When the applied voltage is stable, the positive and negative free charges of *Q* will accumulate on the two plates. As shown in Figure 2 then,

(1) $$\begin{array}{c} Q=CU. \end{array}$$

In the plate capacitor, the capacitance is represented by *C*, and the two poles of the capacitor are pressurized, and the voltage is *U*.

When a solid dielectric material is added between the two poles and pressurized, the amount of positive and negative charges will increase *θ*, as shown in Figure 2, which produces the polarization of the dielectric material. The specific change is caused by the changing external electric field. Eventually, the charge will accumulate on the surface of the plate with the opposite polarity of the charge, which is the result of the positional change of a large amount of free charge along its direction due to the action of the electric field. Leading some of the electric charge in the power supply to the electrode plate, the function is to weaken the effect on the surface electric field, so as to keep the inter-electrode field strength within a certain range [11]. At this time, due to the insertion of a solid dielectric, the power between the plates will increase as follows:

(2) $$\begin{array}{c} Q_{b}=Q+\theta =C. \end{array}$$

And, under vacuum conditions, the electric field between the plates is

(3) $$\begin{array}{c} W=\frac{\gamma }{\lambda }. \end{array}$$

Here, *γ* as the numerator is the charge density, and *λ* as the denominator is the vacuum dielectric constant. The electric field will generate a large amount of polarized charges, which is the result of polarization caused by the air in the middle of the plate electrode being transposed by the insulating dielectric. Among them, the subtraction *γ*^−^ on the numerator represents its density, and the value after the electric field between the plates that is reduced is:

(4) $$\begin{array}{c} W_{1}=\frac{\gamma -\gamma^{-}}{\lambda }. \end{array}$$

According to (3) and (4), the change of the insulating material between the plates leads to a numerical change in the magnitude of the electric field. The ratio of the change is:

(5) $$\begin{array}{c} \frac{W}{W_{1}}=\frac{\gamma }{\gamma -\gamma^{-}}=\kappa . \end{array}$$

Among them, *k* represents the relative permittivity of the dielectric, and its size is only affected by the structure of the dielectric material.

#### 2.2.2. Conductivity of Dielectric

In liquid dielectrics, ions, electrons, and even colloidal particles can be used as carriers in the liquid dielectric, and the difference in carriers is the specific basis for dividing various conductances. Usually, a potential energy diagram can be used to show the state of ion movement, as shown in Figure 3. Suppose the ion is a positive ion, the ion vibrates at the frequency *ƒ*, and the vibration position is at the positions *A*, *B*, and *C* where the energy is the lowest [12].

The ion will be in a stable position in a static state. If the position of the ion is shifted, the kinetic energy of the ion's thermal motion must be greater than the binding barrier of the gravitational force of other ions. If an ion travels along the trajectory from *A* to *B*, the binding force it needs to overcome will decrease by *δ*. If the trajectory is opposite, the binding barrier to overcome will increase by *δ*.

(6) $$\begin{array}{c} \delta =\frac{1}{2}\mu q. \end{array}$$

The impurity ion conductivity is the main conductivity of the pure liquid medium at room temperature. At this time:

(7) $$\begin{array}{c} \eta =\frac{q^{2}\mu v}{6mT}\sqrt{\frac{Sv_{0}}{\omega }}e^{-\left(2u+u_{1}\right)/2mT}. \end{array}$$

As shown in Figure 4, under normal pressure, the constants related to the electric field strength include ion conductivity and electronic conductivity, but sometimes ion conductivity can only be related to the field strength, which only occurs when the applied electric field is not greater than the breakdown electric field strength.

The potential of the particles in the colloid with respect to the liquid is about 0.05 V–0.07 V, and they move in an electric field to form electrophoretic conductance. This is because the colloid particles are also a kind of carriers. The shape of a single colloidal particle is spherical, and the charge quantity *q*=4*ƛϕ*_1_*ϕ*_2_*dU* of the colloidal particle. This migration law is called Walden's law. Under the action of electric field *W*, the electric field force it receives is:

(8) $$\begin{array}{c} F=qW=4ƛ\phi_{1}\phi_{2}dUW. \end{array}$$

Electrophoresis conductivity is:

(9) $$\begin{array}{c} \nu =iq\rho =\frac{8ƛ\;di\;\phi_{1}^{2}U^{2}}{3\alpha },\\ \nu \alpha =\frac{iq^{2}}{6ƛ\;d}=\frac{8ƛ}{3}di\;\phi_{1}^{2}U^{2}. \end{array}$$

In the case where *i*, *d*, *ϕ*_1_, *U* remains unchanged, *ν*, *α* will be a constant.

Apply a high voltage to the liquid medium. At this time, the conductance under a strong electric field is similar to that of a gas medium. The relationship between the current in the medium and the field strength is also similar to that of the gas medium. If the applied voltage is very small, the electric field is weaker. The Ohm's law explains that the current will be positively correlated with the electric field strength. In another case, the conductance has a state of electron impact ionization. In this state, the current and the field strength have an exponential relationship. In this case, only when the electric field is a strong electric field of *W* ≥ 10^7^ V/m.

#### 2.2.3. Loss of Dielectric

The loss of the dielectric is actually composed of two parts, which can be specifically distinguished according to the generation mechanism. But under normal circumstances, the loss will be composed of these two types of loss together, one is polarization loss, and the other is conductivity loss. But for the DC electric field, if the applied voltage does not reach the critical value of partial discharge, the cyclical polarization change process similar to that in the AC field will not occur under the action of the DC voltage, which is the cause of the polarization loss in the medium. When AC voltage is applied, there will be a certain amount of dielectric loss (dielectric loss), which is due to the effect of electrical conduction current and displacement current that converts a part of electrical energy into heat. Dielectric loss is usually not too large, otherwise the insulation will be destroyed due to the temperature higher than the rated value, or even insulation breakdown, which will affect the service life. The main factors affecting dielectric loss are: frequency, temperature, humidity, and field strength.

A new physical quantity dielectric loss tangent value tan  *β* needs to be introduced in the AC electric field. The following formula expresses the amount of loss that occurs when the medium is subjected to an AC electric field after being applied with an AC voltage:

(10) $$\begin{array}{c} Z=UI\;\cos\;\sigma =UI_{P}=UI_{Q}\tan\;\sigma ,\\ Z=U^{2}\varepsilon C_{Z}\tan\;\sigma . \end{array}$$

In the formula, the medium loss angle is represented by *σ*, but the size of tan*σ* has nothing to do with the size of the material sample, but only with the properties of the dielectric itself. In some cases, the value of tan *σ* will increase. For example, excessive environmental humidity will affect the insulation material being damp, or there will be a lot of bubbles and impurities inside the liquid insulation. The greater the tan *σ* value, the greater the dielectric loss of the insulation. Therefore, the physical meaning of the loss tangent value is used to characterize the size of the dielectric loss [13].

### 2.3. Aramid Nanopaper-Based Insulating Materials

Insulating paper is widely used in electrical equipment. Natural cellulose insulating paper is mainly used, and its main component is *α*-cellulose. There are also a small amount of hemicellulose and lignocellulose. Cellulose is a linear polymer substance. Its internal structure is mainly a stable structure formed by the interconnection of hydroxyl and glycoside chains. The hydrogen bonding in the molecule determines the mechanical strength of cellulose. The monomers of lignocellulose and hemicellulose are complex and belong to amorphous polymers, and the interaction between them is relatively small. The polymerization degree of insulating paper commonly used in transformer is generally around 1200. Natural cellulose insulating paper has mechanical properties, good electrical properties, and economic applicability. The use of insulating paper is directly related to the normal use of electrical equipment. The heat-resistant grade of cellulose insulating paper currently used is generally A grade, and its upper limit temperature is generally 105°C [14]. The properties of cellulose insulating paper are shown in Table 1.

Insulating paper will gradually deteriorate due to the effects of temperature, mechanical vibration, and moisture during use, which will cause failures in the use of voltage devices. Temperature is the main factor affecting the use of insulating paper, and the thermal aging of insulating paper directly determines its service life. In addition, when the insulating paper is subjected to high-voltage electricity during use, the insulating paper will experience electrical aging, and the voids and cracks in the insulating paper will cause partial discharges and electrical breakdowns, thus losing its insulation capability. The damage to the performance of the material caused by the oscillating mechanical action of the electrical equipment is called mechanical aging, and the medium in the working environment of the insulating paper damages the material [15].

Aramid has become the fastest-growing new material in the world because of its special high-efficiency properties, and it belongs to the category of aromatic polyamides. Since it was developed and produced by DuPont in the United States in the 1960s, its super-high strength, high modulus and high temperature resistance have been widely recognized [16]. At present, it is mostly used in various cutting-edge fields such as aerospace, military, construction, automobile, machinery, and fields with high material performance requirements.

The aramid fiber formed by resin spinning has an excellent performance and is called “all-round fiber”. Aramid fiber has excellent performance, among which it is famous for its heat resistance, and it also has the advantages of excellent chemical stability, good flame retardancy, and radiation resistance. Aramid has stable performance at high temperatures. Aramid fibers have no glass transition temperature and work for 20,000 hours at 200°C, after which the intensity drops only by about 10%. After continuous use at 300°C for 7 days, the mechanical properties such as strength can still reach more than 50% of the initial value. The strength will be lost when used above 500°C, and carbonization and decomposition will occur above 400°C. Aramid has excellent chemical stability and resistance to various chemical reagents. Aramid fiber has excellent mechanical properties, high strength, high modulus, and large elongation at break. Compared with other products, the breaking strength is high. Its breaking strength can reach 0.47 N/tex, and it has the characteristics of durability and wear resistance [17]. The flame retardant performance of aramid fiber is mainly reflected in its non-flammability in the flame, and it still maintains spontaneous combustion after leaving the flame. The limit oxygen resistance index value is 28%–31%, and the structure is shown in Figure 5.

Aramid resin has excellent electrical properties. The preparation of aramid nanopaper base with aramid resin has a good development prospect in the field of low voltage. There are many types of insulating nanopaper base. Here are a few common insulating nanopaper base for a brief introduction [18, 19]:

1. Polyester nanopaper base is formed by extruding, stretching, blowing, and casting polyester resin. It has the characteristics of high strength, good toughness, good electrical insulation performance, low dielectric loss, and a long-term use temperature of 120°C. Among them, the heat resistance grade of domestic polyester nanopaper base reached *E* grade. Its mechanical properties are excellent, resistant to most chemicals and organic solvents, and low hygroscopicity. Polyester nanopaper base can be directly used as the insulating material of the motor tank, replace the capacitor paper, and be used in the cable.
2. Polyimide nanopaper base, being one of the high-performance nanopaper base, is an indispensable key material in the field of power appliances and microelectronics. It has high temperature resistance, radiation resistance, excellent electrical insulation properties, and good electrical insulation. It has the characteristics of dielectric properties, flame retardancy, and radiation resistance. It is the highest grade electrical insulating nanopaper base used so far, and the heat resistance grade used can reach H grade. Polyimide resin can also be synthesized into 200 grade and 220 grade insulating materials, which is called “golden nanopaper base”.
3. Polypropylene nanopaper base. Polypropylene nanopaper base is widely used in packaging materials. It has good transparency, light weight, outstanding dielectric properties, and low elongation and expansion rates. The long-term working temperature is 100°C, and the price is low. It is widely used in power capacitors and other related equipment.
4. Polycarbonate nanopaper base. Polycarbonate nanopaper base has stable dimensional properties, excellent mechanical properties, good flexibility, low-temperature resistance, high-temperature resistance, high resistance, and low dielectric constant. It is a good insulating material.

### 2.4. Deep Learning

Deep learning is one of the fastest-growing directions in machine learning in recent years. Deep neural network algorithms represented by deep learning have made great achievements in the fields of speech recognition, natural language processing, and image recognition. Its core content is to build an artificial neural network, and through continuous training of large amounts of data to meet a specific demand [20].

Deep learning can be understood in two parts, one is depth, which is to build a multi-layer network to achieve the purpose of depth; the other is learning, using a certain algorithm to update the parameters of each layer until convergence. Deep learning is a supervised learning method. In the learning process, the labels of the training samples and the objectives to be achieved need to be given, and the network parameters of each layer are continuously adjusted to optimize the network performance of deep learning. Deep learning is learning the intrinsic patterns and representational levels of sample data.

## 3. Construction of the Model of the Discharge Mode of the Transformer

### 3.1. Discharging Mode of the Transformer

Due to various defects, the electric field strength of the transformer insulator surface or inside the area appears uneven, when the local breakdown field strength becomes low, partial discharge (partial discharge, referred to as PD) [21] is prone to occur. When partial discharge occurs in the insulation, it affects the insulator life. Generally speaking, due to inaccurate manufacturing processes or irregular installation operations, unbalanced electric field distribution will be generated in the insulating parts of the transformer, forming a phenomenon where electrons are concentrated in a certain part, and the surface of the insulating parts of the transformer will be discharged. On the other hand, during routine maintenance of the transformer, due to the mistakes or unfamiliar techniques of the maintenance personnel, the burrs accidentally touched in the transformer will cause the electric field to deform, which will also cause partial discharge. In addition, the metal parts of the transformer equipment will also discharge after loosening.

Partial discharge of transformer will cause the following hazards:

1. The partial discharge of the transformer will also produce a chemical reaction, and the substances generated by the reaction may damage the insulating parts of the transformer. Insulator damage causes equipment defects, mechanical damage, thermal breakdown, etc.,
2. The temperature of the insulating parts of the transformer rises suddenly, rapidly heats up, accelerates aging, and the performance of the transformer decreases.
3. Brownian motion (the never-ending irregular motion of particles suspended in a liquid or gas) of charged ions is caused, which may break the molecular chains in transformer components.

### 3.2. Transformer Discharge Mode Detection

Due to the different degrees of electric field distortion caused by different insulation aging, different partial discharge modes are produced. There are mainly the following discharges: corona discharge, discharge along the surface, internal discharge, suspension potential discharge. The most important external manifestation of insulation aging is partial discharge. The correct signal detection and reasonable pattern recognition of partial discharge can be used to evaluate the health of the transformer and eliminate dangerous factors early to ensure the safe and stable operation of the transformer. In the process of transformer PD generation, various physical and chemical phenomena such as heat, ultrasound, electromagnetic wave radiation, optics, electric pulse, and gas will appear inside it. Based on related physical and chemical phenomena, a variety of methods for measuring PD signals have been developed [22, 23].

#### 3.2.1. Pulse Current Detection

In the process of partial discharge of the transformer, the transfer of electric charges will occur, and they will form a pulse current in the measuring circuit. This signal can be detected by a current sensor. The pulse current method is widely used in transformer testing and partial discharge experimental research. This method is currently the only standard detection method in the world.

#### 3.2.2. Gas Chromatography

When there is transformer oil and paper age, or when there is an internal failure, many different types of gas will be generated and will be dissolved in the oil in the transformer tank. Different types of gases and differences in gas concentration indicate different types of discharge. The fault state of the transformer is determined by detecting the composition and concentration of the gas in the oil.

#### 3.2.3. Ultrasonic Testing Method

When a partial discharge occurs in the transformer, the molecules around the partial discharge source of the transformer will have a violent impact, and the impact will generate sound waves. This method can be used to detect the position and size of the discharge.

#### 3.2.4. UHF Method

Ultra-high frequency (UHF) method is a new detection method. During the partial discharge of the transformer, there will be very steep current pulses, generating electromagnetic wave signals. At present, many scholars have proved through a large number of experiments that partial discharge can generate electromagnetic waves with very high frequencies, which can reach GHz. The electromagnetic wave excited during the partial discharge of the transformer can be received by the antenna sensor, so that the detection of the electromagnetic signal of the partial discharge of the transformer can be realized.

### 3.3. Discharge Pattern Feature Recognition

As can be seen from Table 2, moment features [24] are often used to characterize image features and describe the distribution of image points. Therefore, different types of PD spectra can be used to generate grayscale images, which can then be used for pattern recognition. The moment information contains many geometric features, such as size, shape, angle, position, etc., Assuming that the two-dimensional discrete function is *f* (*m*, *n*), we calculate *a* + *b* order moment of origin.


(11) $$\begin{array}{c} J_{ab}=\sum_{m}\sum_{n}n^{a}m^{b}f\left(m,n\right). \end{array}$$

If *f* (*m*, *n*) represents the value at the grayscale image (*m*, *n*), then the center of gravity of the grayscale image is

(12) $$\begin{array}{c} \bar{m}=\frac{J_{10}}{J_{00}},\\ \bar{n}=\frac{J_{01}}{J_{00}}. \end{array}$$

The central moment of order *m* + *n* of the gray image is

(13) $$\begin{array}{c} Z_{ab}=\sum_{m}\sum_{n}{\left(n-\bar{n}\right)}^{b}{\left(m-\bar{m}\right)}^{a}f\left(m,n\right). \end{array}$$

The gray-level co-occurrence matrix of the partial discharge gray-level image and the relative gray-level response of neighboring pixels are extracted as the input vector of the support vector machine, and a high recognition rate is achieved.

The measured data based on theoretical analysis and experiments show that the partial discharge signal is a high-frequency signal and the time is extremely short. In the theory based on the discharge mechanism and measurement experiment analysis, four mathematical models are commonly used for simulation of PD pulse signals, formulas (14)–(17) are single exponential decay and double exponential models, single exponential decay oscillation, and double exponential decay [25]. The oscillation model is as follows:

(14) $$\begin{array}{c} f_{1}\left(s\right)=Ue^{-\left(s-s_{0}\right)/\psi }, \end{array}$$

(15) $$\begin{array}{c} f_{2}\left(s\right)=U\left(e^{-1.3\left(s-s_{0}\right)/\psi }-e^{-2.2\left(s-s_{0}\right)/\psi }\right), \end{array}$$

(16) $$\begin{array}{c} f_{3}\left(s\right)=Ue^{-\left(s-s_{0}\right)/\psi }\sin\left(2ƛf_{c}s\right), \end{array}$$

(17) $$\begin{array}{c} f_{4}\left(s\right)=U\left(e^{-1.3\left(s-s_{0}\right)/\psi }-e^{-2.2\left(s-s_{0}\right)/\psi }\right)\sin\left(2ƛf_{c}\left(s-s_{0}\right)\right). \end{array}$$

In the above formula, *U* is the amplitude of the discharge signal, *ψ* is the attenuation constant, *s*_0_ is the start time of discharge, and *f*_*c*_ is the oscillation frequency. Since the partial discharge signal will decay and oscillate during its propagation, the single exponential decayed oscillation model and the double exponential decayed oscillation model are generally used to simulate the signal waveform measured by the experiment.

In the process of discharge signal detection, the transformer is often in operation, which makes the scene noise very loud, but the partial discharge signal is relatively weak, and it is easy to be overwhelmed by noise. The main common types of interference are: periodic narrow-band interference, pulse-shaped interference, and white noise. Among them, the thermal noise of electrical equipment running and the white noise coupled with the line are the most serious. Thermal noise is also referred to as electronic noise, because this noise is generated due to the thermal movement of electrons. White noise is a random signal or random process with a constant power wavelength spectral density.

This article mainly deals with white noise generated by various random noises. The simulation mathematical model is as follows:

(18) $$\begin{array}{c} h\left(s\right)=a•\text{rand}n\left(\text{size}\left(s\right)\right). \end{array}$$

### 3.4. Construction of Transformer Discharge Model

According to the characteristics of insulation defects in the transformer and the location where the discharge occurs, partial discharges are divided into corona discharge, creeping discharge, and insulation internal air gap discharge. Three corresponding electrode structure models are designed in the laboratory as shown in Figure 6, where the thickness of the circular plate electrode is 10 mm and the diameter is 60 mm.

Figure 6(a) shows the needle plate electrode structure, which is used to simulate the corona discharge of transformer insulation. In transformer, insulators are prone to burrs and metal shavings, resulting in uneven field strength and corona discharge. The model is mainly composed of a needle diameter of 0.4 mm, an epoxy plate thickness of 0.8 mm, a diameter of 60 mm, and a circular plate electrode.

Figure 6(b) shows the pole electrode structure, which is used to simulate the creeping discharge of the transformer insulation. It often appears on the high-voltage side, because the field strength formed by it is relatively high, and it is easy to reach the breakdown voltage to form the electric power along the surface. The model is mainly a cylindrical electrode polished by a copper column with a diameter of 10 mm, a thickness of 0.8 mm of epoxy paperboard, and a diameter of 60 mm, as well as a circular plate electrode.

Figure 6(c) shows the air gap structure of the ball electrode, which is used to simulate the internal air gap discharge of the insulation. This is because the insulator is prone to bubbles, impurities, and even cracks during production, and the field strength is relatively concentrated during operation to form internal air gap discharge. The diameter of the ball electrode of this model is 5 mm, the thickness of epoxy paperboard is 0.8 mm, and the diameter is 60 mm. Between the plate electrode and the epoxy paperboard, there is an insulating nanopaper base with a thickness of 0.2 mm and a diameter of 15 mm and a circular plate electrode.

In a closed laboratory environment, use of voltage regulators, transformers, recognizers and other related power electronic components to build a partial discharge experiment platform and circuit is shown in Figure 7. The pulse current method was selected to collect the voltage on the detection impedance and input it to the partial discharge analyzer sampling and saving in TWPD-2E. The sampling frequency is 15 MHz, and the measurement bandwidth is 10 kHz–1 MHz. Among them, each sample under each type of discharge electrode structure model collects data of 50 applied voltage cycles. The specific operation steps are as follows:

1. first, calibrate the entire measurement system, mainly to obtain an accurate apparent charge. Inject a known amount of charge at both ends of the PD model. Assuming that the change in voltage at both ends of the test sample is the same as the change in PD, the injected charge at this time is the PD charge.
2. Measure the maximum allowable experimental voltage of the experimental platform. After the calibration is completed, the calibration device and the partial discharge model are removed from the circuit, and the voltage source is connected to the experimental platform. Without the partial discharge model, the voltage is gradually increased. At this time, the voltage change is recorded. Once the PD pulse appears, Record the value at this time as the maximum allowable experimental voltage *U*_max_ in this experiment.
3. Collect the partial discharge signal, put it into the partial discharge model, and start to increase slowly with a very low initial voltage. Once the discharge pulse appears, the test sample will undergo charge exchange, thereby generating a pulse current in the loop, and detecting and impedance this signal, the voltage at this time can be recorded as the initial discharge voltage *U*_*i*_of the PD model.Increase the voltage to 1.2–1.5 *U*_*i*_so that the input signal amplitude of the signal acquisition system does not exceed 3.5 V as much as possible, and then start sampling. Each sampling records 1000 power frequency cycles, and the sampling interval is 500 power frequency cycles. The results are shown in Table 3.

In this paper, three electrode structure models are Table 3 designed to simulate corona discharge, creeping discharge, suspension discharge, and solid internal air gap discharge; then, the experimental data is collected to generate a three-dimensional spectrum and map it to a two-dimensional spectrum; finally, construct statistics characteristic parameters. A total of 140 sets of data of each type will be collected into 100 sets of training samples, and 40 sets of samples to be identified. They are, respectively, sent to the probabilistic neural network, BP neural network and Hidden Markov model (HMM, Hidden Markov model) to compare and analyze the recognition results of the classifiers. Each classifier needs to perform 15 recognition operations, and the samples are shuffled before each recognition operation to ensure the credibility of the classification results. The highest recognition time and the average time of 15 recognition operations are taken as the evaluation criteria. The result is shown in Figure 8:

The probabilistic neural network is used as a classifier to classify and recognize the three types of transformer discharges, and the recognition effects of BP neural network and HMM are compared. After a large number of experimental simulations, it is found that PNN is better than the other two classifiers in terms of recognition accuracy and recognition time. The results show that using PNN for partial discharge classification and recognition has a good effect.

## 4. Discussion

However, due to the randomness of the PD source and the large amount of noise interference in the detection, the effect of PD pattern recognition in practical applications has not been high [26]. This paper studies the partial discharge models of four artificial transformers,proposes a recognizer based on moment characteristics and probabilistic neural networks, uses genetic algorithms to optimize the smoothing factor of the proposed recognizer, and concludes through experiments and simulations: compared with other neural recognition in the network, PNN performs well in all aspects and responds faster, and the recognition accuracy is not high. Through multiple sets of experimental modeling tests, after eliminating irrelevant data, the accuracy and reliability of the data are maintained within the maximum range. After the introduction of the noise filter processor, PNN will be better used for partial discharge recognition of transformers to ensure the safe use of transformers as much as possible.

## 5. Conclusions

Insulating paper prepared from aromatic polyamide nanopaper has a particularly stable molecular structure with a unique and proper balance of properties. This paper mainly studies the aspects of transformer partial discharge noise denoising, feature extraction, and pattern recognition. Through experiments and simulations, better results have been achieved in the accuracy and time of classification and recognition. But there are also shortcomings. This article does not compare the grayscale image moment characteristics with other PD characteristics. Therefore, other methods can be used to design the characteristics in the next step to find a more suitable transformer partial discharge characteristic. Because the experiment in this paper is based on the offline partial discharge detection in the laboratory, there is little research on the signal denoising part. On-site partial discharge detection is a development trend, and the next step is to study the denoising method of partial discharge signals.

Partial discharge pattern recognition of transformer is a more complicated process. With the development of pattern recognition technology, it is necessary to conduct in-depth research on partial discharge pattern recognition of transformer.

## Figures and Tables

**Figure 1:** Influencing factors of transformer damage.

**Figure 2:** Equivalent polarization circuit diagram.

**Figure 3:** Ion potential energy diagram in liquid dielectric.

**Figure 4:** Ion potential energy diagram in liquid dielectric.

**Figure 5:** Aramid molecular structure.

**Figure 6:** Partial discharge model. (a) Needle plate. (b) Column electrode structure. (c) Ball electrode structure.

**Figure 7:** Circuit diagram of partial discharge experiment.

**Figure 8:** Feature recognition effect of each neural network.

**Table 1:** 500 KV transformer insulation paper performance.

Indicator name			unit	BZZ-075	BZZ-125
Thickness			*µ*m	75 ± 5	75 ± 5
Tightness			g/cm3		0.95 ± 0.05
Tensile strength	Vertical	≧	kN/m	5.80	9.50
	Horizontal	≧		2.70	4.00
Elongation	Vertical	≦	%	6.1	6.9
	Horizontal	≤		2.2	2.5
Common frequency breakdown field strength		≥	kV/mm	8.10	

**Table 2:** Partial discharge signal feature extraction method.

Feature extraction method	Characteristic parameters
Wavelet analysis	Use wavelet to decompose the partial discharge signal, and use the decomposed feature as the feature quantity
Type feature parameters	Extract the fractal dimension of partial discharge gray image and pulse waveform
Statistical feature method	Skewness, kurtosis, number of peak points, discharge pattern factors, phase asymmetry, correlation coefficient, etc.,
Image matrix feature parameters	Extract geometric feature parameters of partial discharge grayscale images
Clustering discrimination algorithm	Extract the waveform characteristic parameters of the partial discharge pulse group

**Table 3:** Experimental data of each model.

Type of discharge	Test voltage	Discharge phase	Apparent charge	The sampling period
Needle plate discharge	7/8/10	240 ∼ 260	160 ∼ 189	1000
Air gap discharge	7/8/10	159 ∼ 176	89 ∼ 98	1000
Creeping discharge	10/12/14	61 ∼ 73	75 ∼ 188	1000
Floating discharge	12/14/18	105 ∼ 136	84 ∼ 97	1000

## Data Availability

The data that support the findings of this study are available from the corresponding author upon reasonable request.
